RETRACTED

# *MiR-130a-3p* inhibits the viability, proliferation, invasion, and cell cycle, and promotes apoptosis of nasopharyngeal carcinoma cells by suppressing BACH2 expression

**DOI:** 10.1042/BSR20160576

**Published:** 2017-06-07

**Authors:** Xin Chen, Bo Yue, Changming Zhang, Meihao Qi, Jianhua Qiu, Ye Wang, Jun Chen

**Affiliations:** Department of Otolaryngology-Head and Neck Surgery, Xijing Hospital, Fourth Military Medical University, Xi’an, Shaanxi Province 710032, China

**Keywords:** BACH2, miR-130a-3p, nasopharyngeal carcinoma

## Abstract

The aim of the present study was to explore the mechanism through which *miR-130a-3p* affects the viability, proliferation, migration, and invasion of nasopharyngeal carcinoma (NPC). Tissue samples were collected from the hospital department. NPC cell lines were purchased to conduct the *in vitro* and *in vivo* assays. A series of biological assays including MTT, Transwell, and wound healing assays were conducted to investigate the effects of *miR-130a-3p* and BACH2 on NPC cells. *MiR-130a-3p* was down-regulated in both NPC tissues and cell lines, whereas BACH2 was up-regulated in both tissues and cell lines. *MiR-130a-3p* overexpression inhibited NPC cell viability, proliferation, migration, and invasion but promoted cell apoptosis. The converse was true of BACH2, the down-regulation of which could inhibit the corresponding cell abilities and promote apoptosis of NPC cells. The target relationship between *miR-130a-3p* and BACH2 was confirmed. The epithelial–mesenchymal transition (EMT) pathway was also influenced by *miR-130a-3p* down-regulation. In conclusion, *miR-130a-3p* could bind to BACH2, inhibit NPC cell abilities, and promote cell apoptosis.

## Introduction

Nasopharyngeal carcinoma (NPC) is a malignant tumor that occurs with high frequency in Southeast Asia and Northern Africa [1]. In 2008, there were an estimated 84400 cases of NPC and 51600 deaths [2]. The major etiological factors of NPC are genetic susceptibility, environmental conditions and Epstein–Barr virus (EBV) infection [1]. It has been reported that certain foods that were high in nitroso compounds and volatile nitrosamines can increase the risk of NPC. It is also connected to lifestyle factors such as smoking [2]. Currently, the most common treatment for NPC is radiation therapy and the 5-year survival rate of stage I and stage II patients treated with radiotherapy has been up to 90% [3]. However, NPC cells can easily invade local tissue or metastasize to remote organs [4]. A recent report showed that the percentage of NPC patients with regional lymph node metastasis and distant metastasis were 74.5 and 19.9%, respectively [5]. The prognoses for stages III and IV patients are still not good, as the 5-year survival rate of patients in these stages ranges from 50 to 70% [3]. Therefore, it is necessary to investigate the molecular bases of NPC metastasis in order to discover new therapeutic approaches.

RETRACTED

MiRNAs are non-protein coding RNA molecules that negatively regulate gene expression by binding to a target sequence in mRNA 3′-UTR at post-transcription level [6,7]. MiRNAs are broadly reported in tumorigenesis and tumor biological processes including differentiation, metastasis, chemoresistance, and tumor development [8]. Plenty of recently published studies have investigated the regulation of miRNA in NPC cells. For example, *miR-205* has been shown to promote the proliferation and invasion of NPC cells; it can also inhibit radiation-induced apoptosis via regulation of PTEN and AKT signaling [9]. On the contrary, *miR-16* has been shown to be a tumor suppressant in NPC cells; it works by targetting fibroblast growth factor 2 (FGF2) in order to inactivate MAPK and PI3K/AKT signaling pathways [10]. The radiosensitivity in NPC cells is also regulated by miRNAs. For instance, *miR-24* [11,12] and *miR-378g* [13] can enhance the radiosensitivity of NPC cells. This provides evidence for a new clinical therapy treatment for NPC that combines radiation therapy with miRNA regulation in order to enhance the effects of treatment. Moreover, prognoses can be predicted based on the measurement of certain miRNA expression levels. Up-regulation of serum *miR-744* has been detected in patients with poor NPC prognoses, and has proven to be an independent factor in the prediction of survival rates [14]. The effects of *miR-130a-3p* were first studied in mice and were later verified in studies with human embryonic stem cells. It appears to be a vertebrate-specific miRNA and is widely developed in angiogenesis, cell cycle, and so on [15]. It has been reported that down-regulation of *miR-130-3p* can promote cisplatin resistance in ovarian cancer cells [16]. Meanwhile, Liu et al. [17] have investigated whether *miR-130-3p* can regulate cell migration and invasion ability by inhibiting Smad4 expression level in gemcitabine-resistant hepatoma cells. Fujita et al. [18] found that *miR-130a* has the potential to be a therapeutic target. These studies have revealed that *miR-130-3p* plays an important role as a regulator in human cancer cells, but the molecular mechanism of *miR-130a-3p* still remains unknown.

BACH2, known as a B-cell tumor suppressor [19], plays a significant role in B-cell maturation, and the regulation of the pre-BCR checkpoint [20]. We have recognized that the balance between BACH2 and BCL6 can maintain the stringency of the GC B-cell repertoire [21], but the mechanism behind this competitive binding behavior by shared target promoters still needs to be investigated [20]. Recently, the oncogenic function of BACH2 has been utilized in several species of malignant tumor. In diffuse large B-cell lymphoma (DLBCL), patients with low expression levels of BACH2 survived longer than those with high expression levels, as BACH2 could be a promising predictor of prognoses for DLBCL [22]. Furthermore, Roychoudhuri et al. [23] reported that BACH2 regulated the function and differentiation of CD8^+^ T cells and other lymphocyte lineages as well as the transcriptional responses to TCR signaling to properly restrict the viral infection. These reports have shown that BACH2 can be a remarkable target gene in cancer suppression. However, the significance of BACH2 in malignant transformation has not yet been determined.

RETRACTED

Here, we analyzed the expression levels of BACH2 and *miR-130a-3p* in NPC tissues and normal nasopharyngeal tissues. We performed the dual-luciferase experiment in order to investigate the underlying regulatory relations between them. Moreover, we transfected *miR-130-3p* mimic and modulated the expression level of BACH2 in NPC cell line CNE. We then determined the comprehensive ability of the different cell groups. We found that BACH2 is a target gene of *miR-130-3p* and that the overexpression of *miR-130-3p* attenuates the promotion effect of BACH2 on NPC cell proliferation, migration, invasion, and anti-apoptosis. Furthermore, tumorigenicity assay in nude mice showed that siRNA effectively inhibited the expression of BACH2 and suppressed the tumor growth *in vivo*.

## Materials and methods

### Human tissue samples

A total of 56 cases of NPC tissues and 45 normal nasopharyngeal epithelial tissue samples were obtained from Xijing Hospital, Fourth Military Medical University. All these specimens were collected between January 2014 and February 2015, and were frozen immediately in liquid nitrogen. The patients agreed to the use of samples and the present study was performed according to the ethical standards of the Ethics Committee.

### Cell culture

Human NPC cell lines CNE, CNE-2Z, S18, HONE-1, C666-1, and human normal cell line NP69 were purchased form the American Tissue Culture Collection (ATCC) and cultured in Dulbecco’s Modified Eagle’s Medium (DMEM) with 10% FBS, 100 U/ml penicillin, and 100 U/ml streptomycin. These cell lines were grown in atmosphere with 95% humidity (37°C and 5% CO_2_) and the medium was replaced every 1 or 2 days.

### RNA extraction and real-time qPCR

Total RNA was isolated from the cell lines and tissues using TRIzol reagent, and was later reverse transcribed into cDNA using a reverse transcription reagent kit (Promega, Madison, WI, U.S.A.). Real-time PCR was performed using a qPCR kit (Invitrogen, Carlsbad, CA, U.S.A.). All the operations were performed in accordance with the manufacturer’s instructions. The primers used in our study were purchased from GeneChem Corporation (Shanghai, China) and the primer sequences are depicted in Table 1.

RETRACTED

**Table 1:** Primer sequences

Gene	Primer name	Sequence (from 5′ to 3′)
*U6*	Reverse transcription	CGCTTCACGAATTTGCGTGTCAT
	Sense	GCTTCGGCAGCACATATACTAAAA
	Antisense	GCTTCGGCAGCACATATACTAAAAT
*miR-130a-3p*	Reverse transcription	GTCGTATCCAGTGCTGGGTCCGAGTGATTCGCACTGG
		ATACGACATGCCCTT
	Sense	TCGTGGGCAGTGCAATGTTAAAA
	Antisense	CAGTGCTGGGTCCGAGTGA
*GAPDH*	Sense	GCACCGTCAAGGCTGAGAAC
	Antisense	TGGTGAAGACGCCAGTGGA
*Bach2*	Sense	CTCGAGAATACCAGCTTGCATGTACCAA
	Antisense	GCGGCCGCTTATCTTCCCGGAATGTGCTTG

### Western blot analysis

Total protein was extracted by lysing the cells in cell lysis buffer. After assessing the protein concentration by BCA protein assay, protein samplse were separated by SDS/PAGE and transferred on to PVDF membranes. The membranes were blocked with 5% non-fat milk at room temperature for 2 h, probed with primary antibodies (1:1000) overnight at 4°C and then washed five times (5 min each time) with PBST/PBS. Membranes were then supplemented with secondary antibodies (1:1500), incubated for 2 h at 37°C and washed for another five times (5 min each time) with PBST/PBS. Finally, band signals were detected with chemiluminescent ECL reagent. All the antibodies mentioned above were purchased from Abcam (Cambridge, MA, U.S.A.).

### Luciferase reporter assay

After synthesizing the wild-type and mutant-type fragments of BACH2, the two fragments were amplified by PCR. The PCR products were then inserted into T4 vector with polyA and transformed in *Escherichia coli* DH5α. The monoclones were used for PCR confirmation. Thereafter, the successfully constructed plasmids and pGL-3 control plasmids (Promega, Madison, WI, U.S.A.) were digested with Xbal restriction enzymes to generate the target fragments, which were then ligated into pGL-3 control vector, respectively. Finally, PCR electrophoresis and DNA sequencing were used to confirm the pGL-3-BACH2 3′-UTR recombinant vector.

The constructed pGL-3-BACH2 3′-UTR plasmids and pRL-CMV plasmids (Promega, Madison, WI, U.S.A.) were transferred into CNE cells, respectively, using Lipofectamine™ 2000. Cells were divided into six groups: pGL-null + mimics negative control, pGL-null + *miR-130a-3p* mimics, pGL-3-BACH2-WT + mimics negative control, pGL-3-BACH2-WT + *miR-130a-3p* mimics, pGL-3-BACH2-MUT + mimics negative control, pGL-3- BACH2-MUT + *miR-130a-3p* mimics. A luciferase assay kit was used, in accordance with the manufacturer’s instructions, to measure the luciferase activity of the cells.

RETRACTED

### Immunofluorescence staining

Cells collected in logarithmic phase were seeded in 24-well plates and divided randomly into three groups, two of which were treated with transfection of mimics negative control and *miR-130a-3p* mimics, respectively. Another group without transfection was set as the control group. After incubating for 36 h, cells were fixed with 4% paraformaldehyde at 4°C for 10 min, rehydrated with 0.5% TritonX-100 for 10 min and blocked in 1% BSA at 37°C for 30 min. Cells were then incubated with primary antibody at 4°C overnight. Cells were then washed with PBS, and incubated with fluorescein secondary antibody at 37°C for 1 h, and washed with PBS again. They were then stained with DAPI, washed with PBS, and blocked in 30% glycerol. Finally, the cells were photographed under a fluorescence microscope.

### Cell transfection

*MiR-130a-3p* mimics (5′-CAGUGCAAUGUUAAAAGGGCAU-3′) and mimics negative control (5′-CAGUACUUUUGUGUAGUACAA-3′) was purchased from Jiaofu Corporation. When the cell confluence reached 80–90%, CNE cells cultured in normal medium were harvested using trypsin. Subsequently, cells were seeded into six-well plates with 2.5 × 10^5^ cells per well and cultured overnight until they reached 40–50% confluence. Finally, cells were transfected with mimics negative control and *miR-130a-3p* mimics (concentration: 50 μM), respectively, using Lipofectamine™ 2000 (Invitrogen).

BACH2 siRNA fragment (5′-GCACACTACAGCGGTCTTA-3′) and NC siRNA fragment (5′-GCAATCGACGGCCTCATTA-3′) were obtained from GeneChem Corporation (Shanghai, China). Cells were seeded into six-well plates (1 × 10^5^ cells/well). When cell confluence reached 40–50%, cells were transfected with siRNA using Lipofectamine™ 2000 (Invitrogen). After 4–6 h, the medium was replaced by normal medium.

To overexpress BACH2, the pCMV-BACH2 recombinant plasmid was constructed using lentivirus vector. The PCR product of BACH2 was inserted into pLVX-IRES-ZsGreen1 vector (Clontech, Mountain View, CA, U.S.A.) and then digested with enzymes between the XhoI and NotI restriction sites. The target fragments collected by a DNA gel extraction kit were taped with T4 DNA ligase. Cells then underwent amplification and DNA sequencing. After the cell confluence reached 80%, 40 µg recombinant plasmids together with 20 µg psPAX2 and 10 µg pMD2G plasmids were transfected into CNE cells by Lipofectamine™ 2000 (Invitrogen). The medium was changed to normal medium after 6 h.

RETRACTED

### Microarray analysis

After transfection with *miR-130a-3p* mimics, cell samples from miR-mimics group and control group were collected for microarray analysis. Total RNA was extracted from frozen NPC tissues or cells using RNA Extraction Kit (Invitrogen, CA, U.S.A.). The Quant-iT RNA Assay Kit (Molecular Probes, Eugene, OR, U.S.A.) was used to detect the RNA concentration. Then, the RNA was hybridized to Human Exon 1.0 ST Arrays (Affymetrix, Santa Clara, CA, U.S.A.) and analyzed as previously described [24].

### MTT cell proliferation assay

Cells collected in logarithmic phase were seeded into 96-well plates (5 × 10^3^ cells/well) and supplemented with corresponding transfection reagents after one night. Each group contained seven parallel wells and a blank control. After cells were incubated at 37°C for 1–5 days, every well of the plates was filled with 10 µl MTT solution (10 mg/ml). Then, 4 h later, 100 µl DMSO was added into all the wells and then absorbance was measured at 570 and 630 nm using ELISA.

### Colony formation assay

Cells of each group were collected and digested with trypsin after 24 h of transfection in six-well plates. Cells were then counted in cell suspension and reseeded in new six-well plates at a density of 600 cells per well. After the plates were placed in the incubator for 10 days and washed with PBS, cells were fixed in 10% methanol for 15 min and stained with Crystal violet for 30 min. Subsequently, cells were washed again with PBS and air-dried. The colony numbers were then counted under a microscope.

### Wound healing assay

We collected CNE cells in logarithmic phase and seeded them into six-well plates (2 × 10^5^ cells/well). After cells had grown to 80–90% confluence overnight, similar sized wounds were scratched on the surface of the wells with 200 µl sterile micropipette tips. The cells were then washed three times with PBS and incubated in DMEM medium with 2% FBS. The migration rate was measured by photographing at three preselected time points (0, 24 and 48 h) under an inverted microscope.

### Transwell invasion assay

After 24 h of transfection, cells were trypsinized and resuspended in DMEM without FBS. As for the transwell chamber, the membrane undersurface was coated with 20 μl of Matrigel (0.5 g/l) and then placed in the chamber at 37°C for 30 min. Subsequently, 200 μl produced cell suspension was added to the upper chamber while the lower chamber was filled with DMEM containing 10% FBS. The transwell chamber was then placed into a 24-well plate. After 36 h of incubation, the chamber was washed, fixed with 4% paraformaldehyde, and stained with 0.1% Crystal Violet. Finally, we photographed the cells under a microscope and counted the number of cells that had passed through the filter membrane in nine random fields.

RETRACTED

### Flow cytometric analysis

The cells in different groups were collected respectively after digesting in 0.25% pancreatic enzymes. The cells were then washed three times with 1× PBS and resuspended with binding buffer. After the number of cells in the cell suspension was counted, the cell density was adjusted to 1 × 10^6^ cells/ml. Then, after being fixed in 70% ethanol at 4°C overnight, cells were collected by centrifugation and subsequently resuspended with 50 mg/ml PI and 50 mg/l RNase. The cell cycle and cell apoptosis were determined by flow cytometric analysis after dark storage at 4°C for 30–60 min.

### Subcutaneous tumor assay

Thirty BALB/c nude mice (SPF grade, 6–8 weeks of age) were randomly divided into five groups (six mice per group). CNE cells (2 × 10^6^) transfected with *miR-130a-3p* mimics, mimics negative control, siRNA-BACH2, and siRNA negative control were injected into the mice of the four groups, respectively. The last group of mice was set as a blank control. The tumor volume was measured every 3 days and calculated using the formula V (mm^3^) = (L × W^2^)/2 (V for tumor volume, L for tumor length, and W for tumor width). On day 23, after cell injection, all the mice were killed to obtain the tumor samples, which were frozen immediately for immunohistochemical analysis.

### Immunohistochemistry

Dissected tissues embedded in paraffin were deparaffinized, rehydrated and antigen retrieved in accordance with the reagent kit instructions. The immunohistochemical staining for sections was observed under a microscope.

### Statistical analysis

Statistical analyses and plotting were performed using GraphPad Prism 6.0 and measurement data were represented as mean ± S.D. Comparisons between the two groups were analyzed by *t* test, while ANOVA was applied for comparisons among multiple groups. *P*<0.05 was considered as statistically significant difference.

## Results

### Expression of *miR-130a-3p* and BACH2 in NPC tissues and cells

To verify the relationship between NPC and *miR-130a-3p*, we detected *miR-130a-3p* expression in NPC tissues and cell samples by RT-qPCR. As seen in Figure 1A,B, the RT-qPCR results showed that *miR-130a-3p* was expressed at an obviously lower level in NPC tissues in comparison with normal nasopharyngeal epithelial tissues. This was consistent in comparison with expression levels of the NP69 cell line (normal cell line), where the expression of *miR-130a-3p* was significantly lower in these NPC cell lines (i.e. CNE, CNE-2Z, S18, HONE-1, and C666-1).

**Figure 1:** *MiR-130a-3p* is down-regulated and BACH2 is up-regulated in NPC cell lines and NPC patients (**A,B**) *MiR-130a-3p* expressions in tissue samples (A) and cell lines (B) were detected by RT-PCR. Normal, normal nasopharyngeal epithelial tissues. (**C,D**). mRNA and protein expressions of BACH2 were detected by RT-PCR (C) and Western blot (D). Data are presented as mean ± S.D. for three independent experiments, ** *P*<0.01, *** *P*<0.001, compared with control.

RETRACTED

Then, we detected mRNA and protein expressions of BACH2 by RT-qPCR and western blot in NPC cell samples. The results (Figure 1C,D) illustrated that the expression of BACH2 was significantly higher in the human NPC cell lines compared with the control group (NP69).

### *MiR-130a-3p* overexpression restrains cell proliferation, migration, and invasion

To explore the effect of *miR-130a-3p* on NPC cells, we transfected CNE cells with *miR-130a-3p* mimics. Cell viability of the CNE cells in the *miR-130a-3p* mimics group was lower than the control group examined by MTT assay (Figure 2B), and the results of colony formation assay in Figure 2C demonstrated that the up-regulation of *miR-130a-3p* suppressed colony formation.

**Figure 2:** Exogenous *miR-130a-3p* attenuated NPC cell viability, cell proliferation, and promoted NPC cell-cycle arrest and apoptosis (**A**) *MiR-130a-3p* expression was detected by RT-qPCR. (**B**) Cell viability of the CNE cells was examined using MTT assays. (**C**) Images and quantitation of colonies of the CNE cells tested by colony formation. (**D,E**) Images and quantitation of the CNE cells determined by cell cycle and apoptosis assays. Data are presented as mean ± S.D. for three independent experiments, *P<0.05, **P<0.01, ***P<0.001, compared with control.

Then, we conducted the flow cytometry to examine the NPC cell cycle distribution, and obtained the results as shown in Figure 2D. The percentage of CNE cells transfected with *miR-130a-3p* mimics in the G_0_/G_1_-phase (68.7%) was significantly higher than that of the control group (55.9%) and that in the S-phase was significantly lower. In addition, the apoptosis rate of CNE cells in the *miR-130a-3p* mimics group (35.83%) was prominently higher than that of the control group (9.1%) (Figure 2E).

The wound healing assay (Figure 3A) demonstrated that the distance between the baselines in the *miR-130a-3p* mimics group was wider than that in the control group. Consistently, in the results of the Transwell assay (Figure 3B), the number of cells that passed through the filter membrane was significantly smaller than that in the control group, suggesting that exogenous *miR-130a-3p* attenuates NPC cell invasion.

**Figure 3:** Exogenous *miR-130a-3p* depresses NPC cell migration, invasion, and NPC growth in mouse xenograft models (**A**) Images of wound healing assays in the CNE cells. (**B**) Images and quantitation of the CNE cells determined by Transwell invasion assays. (**C**) The appearance, total weight, and total volume of tumor samples resected from nude mice with *miR-130a-3p* mimics transfection and control groups. Data are presented as mean ± S.D. for three independent experiments, *P<0.05, **P<0.01, ***P<0.001, compared with control.

RETRACTED

As for the tumor growth *in vivo*, we measured the volume and weight of the tumors resected from the nude mice, and it was observed that tumors in the *miR-130a-3p* group were smaller in size and lighter in weight in comparison with those in the control group (Figure 3C).

### *MiR-130a-3p* directly targets BACH2 in NPC cells

To further investigate the underlying molecular mechanism, we used microarray analysis to find the downstream molecules of *miR-130a-3p*. As shown in Supplementary Figure S1, transfection of *miR-130a-3p* mimics could lead to the dysregulation of many mRNAs. We confirmed these results by detecting the mRNA expressions of S1PR2, Smad4, and BACH2, which were predicted as the targets of *miR-130a-3p* by TargetScan. As S1PR2 and Smad4 have been researched by recent studies [17,25], we chose BACH2 as the research target. As predicted by TargetScan, we found that the 3′-UTR of BACH2 might be the binding site for *miR-130a-3p* (Figure 4A) and we performed the luciferase reporter assay to verify this hypothesis. As shown in Figure 4B, the relative luciferase activity of the pGL-3-BACH2-WT + *miR-130a-3p* mimics group was significantly lower than that of the pGL-3-BACH2-MUT + *miR-130a-3p* mimics group.

**Figure 4:** BACH2 is a direct target gene of *miR-130a-3p* (**A**) Schematic diagram of BACH2 3′-UTR, the corresponding mutant BACH2 3′-UTR and *miR-130a-3p* sequences. (**B**) The relative luciferase activities of CNE in six groups. (**C**) Quantitation of BACH2 protein expression using Western blot in CNE transfected with *miR-130a-3p* mimics as indicated. (**D**) Quantitation of BACH2 protein expression using immunofluorescence in CNE with null, NC, and miR-mimics transfections. BACH2 was visualized using secondary antibodies labeled with Alexa Fluor 594 (red); cell nuclei were stained with DAPI (blue). Data were presented as mean ± S.D. for three independent experiments, ***P<0.001, compared with control.

To further confirm the relationship between *miR-130a-3p* and BACH2, CNE cells were divided into three groups, two of which were transfected with mimics negative control and *miR-130a-3p*, respectively. Another group without transfection served as the control group. Both Western blot and immunofluorescence tests detected the protein expression of BACH2 in CNE cells. The results are displayed in Figure 4C,D. The BACH2 protein expression of the miR-mimics group was significantly less than the Control and siRNA-NC groups.

RETRACTED

### Down-regulation of BACH2 restrains cell proliferation, migration, and invasion

To research the effect of BACH2 on NPC cells, we transfected CNE cells with BACH2 siRNA. As shown by MTT assay in Figure 5B, the cell viability of CNE cells transfected with siRNA-BACH2 was lower than the control and NC groups. Consistently, the colony formation rate was reduced by BACH2-specific siRNA. Both assays demonstrated that the inhibition of BACH2 could attenuate NPC cell proliferation.

**Figure 5:** Inhibition of BACH2 gene expression attenuates NPC cell viability, cell proliferation, and promoted the cell-cycle arrest and apoptosis (**A**) BACH2 expression was detected using Western blot. (**B**) Cell viability of the CNE cells was examined using MTT assays. (**C**) Images and quantitation of colonies of the CNE cells tested by colony formation assay. (**D,E**) Images and quantitation of the CNE cells determined by cell cycle and apoptosis assays. Data are presented as mean ± S.D. for three independent experiments, *P<0.05, **P<0.01, ***P<0.001, compared with control.

The results of the cell-cycle analysis (Figure 5D) illustrated that the number of cells in the G_0_/G_1_-phase in the BACH2-siNRNA group (69.9%) was prominently increased compared with that of the other two groups (both approximately 50%), while the percentage of cells in S-phase was decreased after transfection with BACH2-specific siRNA. The results implied that the cell cycle was arrested by the down-regulation of BACH2 expression in the G_0_/G_1_-phase. The cell apoptosis rate of the CNE cells in the siRNA-BACH-2 group was significantly higher (45.6%) than that in the control groups (both approximately 10%). This suggested that the inhibition of BACH2 expression could accelerate cell apoptosis.

As we can see in the results of the wound healing assay (Figure 6A), the distance between two baselines in the siRNA-BACH2 group was wider than that in the other two groups, which suggested that suppressing the expression of BACH2 repressed NPC cell migration. Additionally, the results of the Transwell assay (Figure 6B) showed that the number of cells that passed through the filter membrane was obviously lower than in other groups. This result indicated that inhibition of BACH2 suppressed cell invasion.

**Figure 6:** Inhibition of BACH2 gene expression depresses NPC cell migration, invasion, and tumor growth (**A**) Images of wound healing assays in the CNE cells. (**B**) Images and quantitation of the CNE cells determined by Transwell assays. (**C**) The appearance, total weight, and total volume of tumor samples resected from nude mice with BACH2 siRNA transfection and control groups. (**D**) The expression of BACH2 protein was detected by immunohistochemistry using specific antibodies. (**E**) The results of Western blot showed that enhanced BACH2 gene expression attenuates the regulation ability of *miR-130a-3p* on the expression of epithelial–mesenchymal transition (EMT)-associated genes in CNE. Data were presented as mean ± S.D. for three independent experiments, ***P<0.001, compared with control.

RETRACTED

Furthermore, when we measured the tumor weights and tumor sizes of the samples obtained from the nude mice, we found that the tumors in the siRNA-BACH2 group were smaller in size and lighter (in weight) in comparison with the control groups (Figure 6C). This suggested that down-regulation of BACH2 restrained tumor growth *in vivo*. In the results of the immunohistochemistry in Figure 6D, it was confirmed that the protein expression of BACH2 in the tumor samples was successfully decreased by the siRNA.

### BACH2 overexpression reduces the effect of *miR-130a-3p* on suppressing the EMT procedure

Cells were divided into five groups: control, mimics negative control, *miR-130a-3p* mimics, *miR-130a-3p* mimics + pCMV and *miR-130a-3p* mimics + pCMV-BACH2. The protein expression of EMT-associated genes was detected by Western blotting and the results are shown in Figure 6E. After transfection of *miR-130a-3p* mimics, E-cadherin expression was increased while the expression of Vimentin and N-cadherin were decreased. When *miR-130a-3p* and BACH2 expression were up-regulated simultaneously. However, the expression of E-cadherin was decreased and the expression of Vimentin and N-cadherin were increased in comparison with the *miR-130a-3p* mimics + pCMV group.

## Discussion

MiRNAs have been reported to play an important role in NPC and its prognosis [26,27]. Several miRNAs were investigated as tumor suppressors by targetting different proteins or signaling pathways, such as *miR-34b* [1], *miR-34c* [28], *miR-133b* [29], *miR-223* [4], and *miR-497* [30]. Some studies have found *miR-130-3p* to be significantly down-regulated in several cancers. Ouyang et al. [31] found that *miR-130-3p* was down-regulated in triple-negative breast cancer (TNBC) compared with matched peritumoral counterparts; Ottley et al. [32] observed that *miR-130-3p* significantly decreased in activin-sensitive prostate cancer (LNCaP) cells; and Snyder-Talkington et al. [33] claimed that *miR-130-3p* was down-regulated in bronchioloalveolar adenocarcinoma. The present study found that *miR-130a-3p* was expressed at a lower level in NPC tissues than normal tissues, and that the expression level of NPC cell lines also coincided with the results in tissues. The down-regulation in NPC tissues matched the trend in previous reports and showed the possibility of *miR-130a-3p* as a tumor-suppressing miRNA. The overexpression of *miR-130a-3p* showed an inhibitory effect on migration and invasion of human liver cancer cells HepG2 [17]. Meanwhile, *miR-130a* was highlighted in HCC drug resistance and progression [34,35]. In the present study, the proliferation ability of NPC cell line CNE was inhibited by up-regulated *miR-130a-3p*. Pan et al. [36] discovered that *miR-130a* directly targetted RAB5A to inhibit the migration and invasion of human breast cancer cells. Consistent with these results, our *in vitro* as well as *in vivo* studies also showed that overexpression of *miR-130a-3p* promoted the invasion, migration as well as proliferation of NPC cells. We thus speculated that *miR-130a-3p* might be a suppressor of NPC tumors.

RETRACTED

Meanwhile, in the past few years, there have been many reports proposing that BACH2 is an important factor in numerous autoimmune diseases, in lymphoid-specific transcription, and in B-cell development [19,37]. However, the results have shown a totally different function of BACH2 in tumor growth. Sakane-Ishikawa et al. [38] reported that a high expression level of BACH2 showed better DFS and OS rates in DLBCL. In contrast, Ichikawa et al. [22] found that patients with low expression levels of BACH2 could survive longer with the same kind of tumor. Until now, there has been no report dedicated specifically to the investigation of BACH2 expression levels in NPC cells. Our study showed that BACH2 was overexpressed in a variety of NPC cell lines as compared with normal cells, and that there was a similar trend at the protein level. We also found that low expression of BACH2 greatly inhibited the proliferation of NPC cells while also inhibiting their invasion and migration. In the nude mice tumor formation experiment, the tumor growth rate in mice with low levels of BACH2 decreased significantly. The reason for that might be that BACH2 was promoting tumor immunosuppression. Roychoudhuri et al. [39] researched whether BACH2 could promote the growth of tumors by Treg-mediated inhibition of CD8^+^ T cells as well as concomitant IFN-γ-dependent effector mechanisms in melanoma and lymphoma. Based on the experimental result of BACH2-deficient mice, he claimed that BACH2 was required in establishing immunosuppression in CD4^+^ T cells and potently inhibited the activity of CD8^+^ T cells, which are also antitumor cells.

RETRACTED

EMT is a biological process during which epithelial cells lose their epithelial morphology, increase their ability of invasion, migration, and apoptosis resistance to assume a status as mesenchymal cells [40,41]. It is widely accepted that EMT process is vital in the invasion as well as metastasis of malignant tumors [41]. Moreover, by simultaneously overexpressing BACH2 and *miR-130a-3p* in NPC cells, we discovered the regulatory function of this miRNA. The preceding results of our experiment showed that BACH2 enhanced the migratory as well as invasive ability of NPC cells, while *miR-130-3p* inhibited these capabilities, which implied that they might be involved in the EMT process. During the EMT process, epithelial cells lose their polarized organization and cell–cell junctions, gain the mesenchymal markers as a fundamental change in cellular morphology and phenotype, and thus improve their capacity for migration and invasion, resulting in tumor aggressiveness [42–44]. EMT has been recognized as an important role in cancer cell metastasis [45]. During the enhancement of EMT process, the expression of the epithelial markers such as β-catenin and E-cadherin are reduced, whereas the mesenchymal markers, for instance Vimentin and N-cadherin are increased. This can then promote the migration and invasion of cancerous cells [42]. In our study, the expression levels of β-catenin and E-cadherin increased when *miR-130a-3p* was up-regulated, while Vimentin and N-cadherin showed lower expression levels. However, the overexpression of BACH2 could weaken the inhibitory effects of *miR-130a-3p* in EMT process of NPC cells.

In summary, the present study demonstrated that *miR-130-3p* could be an NPC tumor suppressor and repress the EMT process in NPC cells. The interaction of *miR-130-3p* and BACH2 might be applied in clinical treatment for NPC patients. However, the specific path of EMT process influenced by BACH2 has not yet been determined, thus further investigation is required.

## Abbreviations

DLBCL: diffuse large B-cell lymphoma
DMEM: Dulbecco’s Modified Eagle’s Medium
EMT: epithelial–mesenchymal transition
NPC: nasopharyngeal carcinoma
